# Research on the Health Literacy Status and Compliance Behavior of Patients with Acute Coronary Syndrome

**DOI:** 10.1155/2021/9648708

**Published:** 2021-11-08

**Authors:** Huanya Liu, Jing shen, Sien Li, Ying Song, Mingfei Ju

**Affiliations:** ^1^Emergency Department, Affiliated Hospital of Chengde Medical University, Chengde Hebei 067000, China; ^2^Internal Medicine-Cardiovascular Department, Affiliated Hospital of Chengde Medical University, Chengde Hebei 067000, China

## Abstract

This study is aimed at assessing the current status of ACS patients' health literacy and medication compliance, analyzing the relationship between the two, and providing ideas for clinically improving the medication compliance of ACS patients and preventing the recurrence of cardiovascular events. ACS patients need long-term medication to prevent vascular restenosis after surgery, and bad living habits and mood swings will affect postoperative recovery, so clinical interventions are needed to help patients establish a healthy lifestyle. The effect of conventional care is not ideal. Therefore, this paper uses regression analysis to analyze the correlation between the health literacy status of ACS patients and the compliance behavior, combines the investigation and experiment to perform regression analysis and uses mathematical statistics to process data. The connection between health literacy level and compliance behavior is discovered via a study, providing a point of reference for future research.

## 1. Introduction

Cardiovascular disease is now the most common illness in the world, and it is on the rise in our nation year after year. Cardiovascular disease is the leading cause of mortality among the different causes of death. Every year, more than 15 million individuals worldwide die from cardiovascular disease [1]. According to World Health Organization data, cardiovascular disease and its consequences, particularly heart failure following ischemia, are expected to become the leading cause of disability and death globally by 2020. Furthermore, it is becoming more common as people become older. The China Cardiovascular Disease Report 2016 shows that cardiovascular disease has become the number one cause of death among urban and rural residents in my country, and the proportion in rural areas is 44.8% and that in urban areas is 41.9%. According to the registration in the report, there are about 290 million patients with cardiovascular disease in the country, of which 270 million are hypertension patients, 4.5 million patients with heart failure, 2.5 million patients with myocardial infarction, and at least 7 million patients with stroke. The data shows that the rising trend of cardiovascular mortality is mainly due to the rising mortality of coronary heart disease. At the same time, data shows that China's cardiovascular mortality rate is significantly higher than that of Western developed countries. If effective prevention and treatment measures are not taken, it is estimated that between 2010 and 2030, the number of cardiovascular events in China will increase by 21.3 million, and the number of deaths will increase by 7.7 million. This will cause serious harm to the patient's health and life and put a heavy economic burden on the patient's family and society [2]. The burden of cardiovascular disease is increasing and has become a major public health problem. It is urgent to prevent and treat cardiovascular disease. Common risk factors for coronary heart disease include old age, men and postmenopausal women, smoking, hypertension, diabetes, hyperlipidemia, abdominal obesity, and family history of early-onset coronary heart disease. In China, there are presently 270 million people with hypertension, and hypertension awareness, treatment, and control rates are still extremely low among the general population [3].

According to the 2010 Global Adult Tobacco Survey (GATS) China Project report, there are 356 million smokers over 15 years old, and the number of passive smokers is even more, which is 738 million. In the 2010 national survey, the prevalence of hypercholesterolemia in men and women over 18 years old was 3.4% and 3.2%, respectively, and the prevalence of hypertriglyceridemia in men and women is 13.8% and 8.6%, respectively [4]. Among the 12,040 dyslipidemia patients surveyed nationwide in 2013, only 39% of the patients received lipid-lowering treatment, most of them used statins, and the low-density lipoprotein cholesterol compliance rate was only 25.8%. The prevalence of diabetes in China is 11.6%, but the treatment rate is only 25.8%, and the treatment compliance rate is only 39.7%. These data are not optimistic. Coronary atherosclerotic heart disease (CHD) refers to a heart disease caused by atherosclerosis of the coronary arteries, which causes stenosis or obstruction of the lumen and leads to myocardial ischemia, hypoxia, and even necrosis [5]. It is referred to as coronary heart disease, also known as ischemic heart disease (IHD). It is also the most frequent kind of atherosclerosis, which causes organ lesions, as well as a common disease that puts people's health at danger. Acute coronary syndrome (ACS) is a kind of coronary artery disease that may cause arrhythmia, heart failure, and even death. ACS is classified as ST segment myocardium infarction (STEMI), non-ST segment myocardium infarction (NSTEMI), and unstable angina pectoris based on the characteristics of the chest pain, the ECG performance of the chest pain, and whether or not the indicators of myocardial necrosis are positive (UAP). The pathological foundation of coronary atherosclerotic plaque rupture or invasion, due to full or partial occlusive thrombosis, is the pathological basis of ACS. Furthermore, a significant number of investigations have shown that the major pathophysiological processes of ACS include coronary atherosclerotic plaque rupture, vasospasm, and subsequent platelet adhesion, aggregation, and secondary thrombosis. The traditional definition of coronary heart disease is caused by an imbalance of myocardial oxygen supply based on coronary atherosclerosis. With the development and popularization of coronary angiography and intravascular ultrasound, we have found that some ACS are not completely secondary to unstable plaque rupture or thrombus formation. It has been reported in the literature that about 6% of patients with acute myocardium infarction (AMI) showed no vulnerable plaque formation and rupture in coronary angiography intravascular ultrasound. These patients are often younger at onset and often have no related high-risk factors for coronary heart disease [6, 7].

This article investigates the health literacy level and compliance behavior of patients with acute coronary syndromes, focusing on scientific and effective treatment techniques and nursing methods, as well as effective theories for the treatment and rehabilitation of acute coronary syndromes.

## 2. Related Work

Clinically, about 20% of patients with acute coronary syndromes have atrial fibrillation, which is associated with reduced left ventricular ejection fraction and age [8]. In addition, these patients often have a history of chronic diseases such as hypertension and diabetes, and the results of coronary angiography often show diffuse multivessel disease. Studies have confirmed that patients with acute coronary syndrome and atrial fibrillation have a significantly higher risk of adverse cardiovascular events such as malignant arrhythmia and heart failure than patients with simple acute coronary syndrome [9]. The literature [10] also showed that the short-term and long-term mortality of patients with acute coronary syndrome and atrial fibrillation increased by 20% and 34%, respectively. Patients with acute coronary syndrome and atrial fibrillation have complex conditions, contradictions in treatment, and poor short-term and long-term prognosis [11].

In my nation, the age distribution of coronary heart disease is now dominated by the elderly. A number of studies have shown a link between age and the risk of acute myocardial infarction [12]. According to the literature [13], the older a patient is when they have an acute myocardial infarction, the less likely they are to have the usual pain symptoms. From this perspective, it seems that the patient's perception of the sickness deteriorates with age, which may be a protective element in the patient's psychological adaption to the condition. Coronary heart disease is more common among the elderly. On the one hand, many illnesses, a lack of financial resources, and a lack of family companions lead patients to urgently need social family assistance. They do not, however, have these supports, and this discrepancy is likely to have an effect on patients' psychological adaption. The anxiety and depression of patients with acute myocardial infarction were examined in the literature [14], and it was shown that older individuals are more prone to anxiety and sadness. Low education, dread of illness, and fear of recurrence are all linked to anxiety and sadness in older individuals with acute myocardial infarction. Literature [15] found that elderly patients with acute myocardial infarction and young patients have different degrees of psychological problems. The main cause of anxiety in elderly patients is suffering from multiple complications, worrying about a poor prognosis, and having sleep disorders. Impatience, irritation, a lack of patience, usual physical symptoms, and fear that the illness may impact family and job are the major causes of anxiety among young patients.

### 2.1. Method

In this study, 280 ACS patients were enrolled in the study from the hospital, and they all signed the informed consent form. The general data survey scale uses the general data survey scale self-made in the hospital, which includes gender, age distribution, occupation, education level, family income, and health knowledge acquisition channels. Moreover, this paper collects disease-related data of ACS patients, including body mass index (BMI), heart disease history, number of hospitalizations, course of disease, degree of coronary artery disease, and revascularization [16].

All investigators in this study are trained and qualified. The questionnaire was distributed and collected on the spot. Patients should be informed about the study's aim and procedures, as well as any confusing questions, by questionnaire investigators. They cannot, however, utilise inductive or suggestive language, nor can they check for missing elements and add them in a timely manner. Two medical statistics experts are in charge of data input and verification once the questionnaires have been gathered.

The purpose of this essay is to look at medication compliance as a key component of compliance behavior. In addition, the statistical information acquisition ability, communication and interaction ability, willingness to improve health, willingness to receive financial support, and total score of health literacy are used as the main reference indicators for examining the relationship between patients' health literacy and compliance behavior, and the results are counted .

## 3. Result

The logistic multifactor analysis affecting the health literacy of ACS patients is shown in Table 1 and Figure 1.

The statistics of patients' medication compliance and health literacy status are shown in Tables 2–6 and Figures 2–6.

## 4. Analysis and Discussion

Most patients with ACS have health knowledge and attitudes but lack the capacity to translate these into healthy habits and skills, according to one research. Furthermore, due to a variety of reasons, the health literacy level of ACS patients is not encouraging. The findings of most research show that age is a risk factor that influences the health literacy of patients with ACS. The reason may be that the older the patients are, the more they emphasize their own experience and reject new things and ideas. Therefore, even if they have the desire to learn actively, due to the decline of physical skills, cognition, understanding, and action ability, there are many difficulties in mastering health knowledge and practicing healthy behaviors. Therefore, the health promotion ability is low. However, most of the career families of patients under the age of 50 are at the peak period, and they can use their own personal networks or various media to obtain health-related information, knowledge, and skills to maintain their own health. This study shows that the higher the level of education, the higher the health literacy, which is consistent with the conclusions of a large number of studies. The main reason is that people with a higher education level have significantly higher access to health resources and attitudes than those with a relatively low level of education, and they have relatively strong restraint and control over unhealthy behaviors, and they pay more attention to their own health management capabilities. People with lower educational levels, on the other hand, have worse reading and comprehension abilities and are unable to interact effectively with medical personnel, resulting in more misunderstanding regarding their own health habits as well as illness diagnosis and treatment. Even some patients have negative emotions, which seriously hinders the effective development of treatment work and is not conducive to timely and effective treatment. This result also suggests that health education is a strong tool for promoting health literacy in patients with ACS and that it can significantly enhance patients' health literacy levels. This study shows that the history of heart disease can significantly affect the health literacy of patients. The reason may be that patients with a history of heart disease have a certain degree of knowledge about heart disease. As a result, they have a higher degree of awareness of ACS-related symptoms and prevention, a more positive attitude, and a higher health literacy ability. This study shows that the more severe the coronary artery disease, the lower the level of health literacy. The reason for the analysis is that patients with severe coronary artery disease have limited ability to obtain health information, leading to insufficient confidence in coping with the disease. However, people with low health literacy usually have resistance to health behaviors, leading to further deterioration of the disease. This indicates that patients with severe coronary artery disease should be aware of their health literacy level and that healthcare providers should assist patients understand the significance of health literacy in the illness's outcome.

This study shows that the history of revascularization is the main factor that affects the health literacy of patients with ACS. The reason is that patients who have undergone a history of revascularization have improved disease awareness to a certain extent and have a higher desire for health information and are more sensitive. At the same time, patients undergoing revascularization are often in serious illness. After experiencing this pathological process, patients are more aware of the importance of healthy behaviors, so they can adhere to reasonable diets, compliance behaviors, etc. and have a higher level of health literacy.

ACS patients' medication adherence has to be improved. ACS patients should be treated with secondary preventive medicines if there are no obvious contraindications, according to current domestic and international recommendations, independent of their pathological type or whether they need stent intervention. Medication compliance is an important outcome factor for evaluating the prognosis of ACS patients since secondary preventive pharmacological therapy is necessary to minimise the recurrence of unfavourable cardiovascular events in ACS patients. This group of patients had a medication noncompliance rate of 68.52 percent, indicating that more than two-thirds of ACS patients had poor drug compliance. The present state of drug compliance among ACS patients is said to be concerning. The percentage of patients who forgot to take medicine and who discontinued taking medication after their symptoms improved was quite high among the four issues of medication noncompliance. The following may be the reason: (1) ACS patients often require combination medication. Although epidemiology has shown that the population of ACS patients tends to be younger, this group is still dominated by middle-aged and elderly people. Moreover, middle-aged and elderly patients often have a decline in their understanding and recognition of drug information, which affects their medication compliance. (2) The patient has insufficient understanding of the significance of secondary preventive drug treatment and prevention of cardiovascular events, or due to financial constraints and other factors, the drug is discontinued without authorization when the symptoms are relieved. (3) The low level of medication literacy of ACS patients directly affects medication compliance. In clinical practice, for forgetting to take medication, we can use smart portable devices based on smart medical care, such as “Internet +” to remind patients to take medication regularly, or form a multidisciplinary cooperation model including pharmacists to conduct comprehensive interventions. Nurses may also use innovative forms of health education, such as APP software and a WeChat official account, to raise patient knowledge of the need of sticking to secondary preventive medicine. Simultaneously, we may dig deeper into the precise causes for patients' noncompliance behavior in order to offer more focused nursing solutions.

The health literacy of ACS patients needs to be improved. After studying the health literacy status of patients with cardiovascular disease, it is found that it is closely related to the patient's prognosis. The health literacy level of patients with acute myocardial infarction is similar, showing a low level. Patients with low health literacy have a poor understanding of disease knowledge, and their ability to screen, acquire, and absorb health knowledge is also limited, which affects their self-management ability. Therefore, we recommend that clinical nurses take the following measures: (1) the evaluation and reevaluation of health literacy can be incorporated into the clinical nursing work of ACS patients to explore the influencing factors of health literacy and formulate intervention plans. (2) Medical staff can produce ACS disease-related knowledge and first aid education manuals that are both illustrated, easy to understand, and popular. In particular, it is necessary to highlight the identification of typical and atypical symptoms, the timely dosage of nitroglycerin, the interval time, the total amount taken, and the best way of prehospital first aid. (3) It is necessary to rely on the medical consortium and the “Internet +” platform to build a continuous care method and increase the popularization rate of disease common sense and first aid knowledge among the discharged ACS population, thereby improving the health literacy of patients.

## 5. Conclusion

This study shows that ACS patients with low health literacy have worse compliance with medication. Moreover, patients with low health literacy may have varying degrees of difficulty in reading drug labels and understanding drug side effects and drug prescriptions. The resulting unsafe medication situation will lead to unsatisfactory medication treatment and affect medication compliance. Patients with low health literacy have difficulty understanding drug-related information such as drug usage, dosage, and indications. Their real drug use may differ from what the medical system records. Furthermore, some study findings suggest that health literacy refers to the information and abilities needed for optimal drug adherence. Nurses are reminded that when it comes to increasing medication compliance, the impact of the variable of health literacy should not be overlooked. They can first evaluate and improve the health literacy level of ACS patients and then improve medication compliance on this basis.

The medication compliance and health literacy level of ACS patients need to be improved urgently. Therefore, clinical nurses should pay attention to evaluate and improve the health literacy level of ACS patients and then improve their medication compliance. However, this study did not analyze in detail the influencing factors that lead to unsatisfactory medication compliance and health literacy of ACS patients and did not pay attention to ACS patients at different periods or discharged from the hospital, which needs to be verified in future studies.

## Figures and Tables

**Figure 1:** Regression analysis of health literacy status.

**Figure 2:** Visual display of results of information acquisition capabilities.

**Figure 3:** Visual display of the results of communication and interaction capabilities.

**Figure 4:** Visual display of results of willingness to improve health.

**Figure 5:** Visual display of the results of economic support willingness.

**Figure 6:** Visual display of the results of the total score of health literacy.

**Table 1:** Logistic multifactor analysis affecting the health literacy of ACS patients.

Risk factors	*B*	SE	Wald*χ*^2^	95% CI	*P*
Age	0.63529	0.26967	5.6055	1.89476	1.682-6.265
Education level	0.75447	0.32421	5.46915	2.13211	1.265-3.618
History of heart disease	1.2625	0.42218	6.1913	2.81487	1.18-4.986
Degree of coronary artery disease	1.34128	0.38178	12.46542	3.81073	1.137-9.652
History of revascularization	0.92213	0.28987	10.2212	2.51692	1.359-6.488

**Table 2:** Statistics of the results of information acquisition capabilities.

Number	Value	Number	Value	Number	Value
1	45.47	21	53.65	41	52.61
2	44.36	22	55.51	42	48.54
3	42.59	23	55.99	43	51.30
4	43.46	24	41.41	44	47.08
5	52.58	25	43.27	45	48.47
6	51.97	26	52.31	46	47.54
7	42.00	27	39.60	47	47.76
8	51.83	28	52.55	48	53.53
9	45.33	29	46.67	49	47.11
10	44.24	30	55.94	50	43.04
11	45.10	31	39.43	51	48.86
12	45.42	32	55.58	52	55.64
13	44.62	33	48.68	53	41.19
14	45.16	34	39.10	54	46.88
15	47.65	35	46.44	55	55.09
16	39.17	36	46.92	56	41.16
17	43.72	37	40.81	57	48.69
18	40.00	38	44.83	58	44.89
19	47.67	39	54.63	59	46.46
20	40.16	40	46.85	60	41.07

**Table 3:** Statistics of the results of communication and interaction capabilities.

Number	Value	Number	Value	Number	Value
1	55.33	21	47.52	41	51.05
2	50.20	22	52.09	42	56.98
3	47.35	23	55.48	43	58.65
4	52.22	24	51.55	44	54.05
5	55.88	25	56.98	45	48.40
6	45.25	26	53.06	46	46.18
7	53.95	27	56.37	47	52.01
8	54.87	28	55.80	48	49.47
9	48.28	29	54.33	49	57.91
10	50.57	30	45.76	50	58.58
11	60.31	31	46.70	51	58.35
12	60.74	32	53.32	52	49.21
13	53.80	33	53.82	53	60.31
14	56.97	34	49.56	54	55.37
15	58.05	35	46.18	55	58.41
16	56.81	36	57.11	56	45.08
17	48.77	37	60.56	57	57.39
18	59.42	38	48.04	58	51.59
19	59.38	39	57.79	59	49.55
20	55.21	40	57.31	60	55.90

**Table 4:** Statistics of results of willingness to improve health.

Number	Value	Number	Value	Number	Value
1	78.19	21	81.36	41	81.82
2	82.83	22	82.18	42	73.83
3	87.41	23	85.07	43	61.13
4	77.52	24	65.73	44	75.31
5	72.82	25	73.90	45	80.56
6	77.07	26	69.48	46	67.03
7	86.73	27	78.68	47	75.83
8	83.28	28	70.38	48	73.16
9	69.58	29	68.06	49	70.37
10	86.41	30	63.71	50	74.39
11	80.73	31	70.17	51	65.91
12	83.47	32	62.12	52	74.52
13	73.46	33	71.93	53	68.62
14	69.69	34	71.26	54	64.20
15	75.68	35	63.13	55	85.59
16	77.65	36	76.37	56	61.26
17	86.28	37	67.73	57	80.30
18	71.55	38	83.17	58	63.49
19	80.61	39	81.02	59	82.12
20	81.00	40	69.59	60	86.77

**Table 5:** Statistics of the results of financial support willingness.

Number	Value	Number	Value	Number	Value
1	45.78	21	52.08	41	38.34
2	50.20	22	50.20	42	42.01
3	38.16	23	53.98	43	53.78
4	44.67	24	53.75	44	55.41
5	45.27	25	51.71	45	56.02
6	42.89	26	44.04	46	53.93
7	50.12	27	50.45	47	39.80
8	56.91	28	46.42	48	38.79
9	42.85	29	45.08	49	48.05
10	55.16	30	47.26	50	41.67
11	45.01	31	53.90	51	46.54
12	40.50	32	44.80	52	49.28
13	53.09	33	39.69	53	46.69
14	45.74	34	45.15	54	49.45
15	56.07	35	42.23	55	52.28
16	42.26	36	55.54	56	38.40
17	53.90	37	41.26	57	40.29
18	38.26	38	42.41	58	49.95
19	49.30	39	54.95	59	38.48
20	55.32	40	48.96	60	55.49

**Table 6:** Statistics of the results of the total scores of health literacy.

Number	Value	Number	Value	Number	Value
1	70.40	21	52.24	41	70.30
2	71.96	22	55.13	42	50.47
3	62.28	23	57.08	43	66.23
4	67.36	24	71.41	44	55.38
5	49.88	25	64.06	45	51.32
6	67.71	26	50.92	46	52.77
7	51.61	27	71.01	47	56.34
8	59.14	28	66.93	48	69.92
9	50.78	29	71.78	49	55.94
10	56.18	30	68.13	50	53.33
11	49.82	31	64.73	51	59.86
12	62.66	32	54.33	52	71.16
13	58.79	33	55.33	53	52.38
14	68.96	34	66.26	54	62.80
15	62.45	35	71.46	55	60.87
16	66.28	36	68.58	56	63.28
17	52.95	37	67.38	57	54.08
18	51.10	38	54.36	58	67.63
19	66.15	39	65.62	59	55.52
20	64.66	40	50.17	60	59.56

## Data Availability

The data used to support the findings of this study are included within the article.
